This article has been retracted.

# EF-Hand Domain-Containing Protein D2 (EFHD2) Correlates with Immune Infiltration and Predicts the Prognosis of Patients: A Pan-Cancer Analysis

**DOI:** 10.1155/2022/4878378

**Published:** 2022-03-15

**Authors:** Yu Wang, Meiqi Song, Binbin Gao

**Affiliations:** ^1^Nanjing Medical University, 211103, China; ^2^Haerbing Medical University, 150076, China

## Abstract

**Background:**

EF-hand domain-containing protein D2 (EFHD2) has recently been reported to participate in initiation of cancer. More evidence indicates that EFHD2 plays an important role in tumors, but the pan-cancer analysis of EFHD2 is still very limited.

**Methods:**

In this study, we downloaded the original mRNA expression data and SNP data of 33 kinds of tumor data. The gene expression data of different tissues were downloaded from the GTEX database, combined with TCGA data and corrected to calculate the difference of gene expression. The data of total survival time (OS) and progression-free survival (PFS) of TCGA patients were downloaded from the Xena database to further survey the relationship between the EFHD2 expression and prognosis. The CIBERSORT algorithm was used to analyze the RNA-seq data of 33 kinds of cancer patients in different subgroups. In this study, NCI-60 drug sensitivity data and RNA-seq data were downloaded to explore the relationship between genes and common antineoplastic drug sensitivity through correlation analysis. In this study, GSEA analysis was carried out from the Molecular Signature database through the packages of “clusterprofiler” and “enrichplot.” By comparing the differences of signal pathways between high and low gene expression groups, the possible molecular mechanism of prognostic differences among 33 kinds of tumors was determined.

**Results:**

Our results indicated that EFHD2 was highly expressed in 23 kinds of tumors. In addition, EFHD2 was associated with stage in many kinds of tumors. The expression of EFHD2 was closely related to the OS of 12 kinds of cancer patients. In addition, Kaplan-Meier- (KM-) plot survival analysis indicated that the high expression of EFHD2 was related to the poor OS of 5 kinds of cancer, and the expression of EFHD2 was closely related to the PFI of 5 kinds of cancer patients. The expression of EFHD2 was closely related to immune infiltration, among which 18 cancers were significantly correlated with CD8T cells, 14 cancers were significantly correlated with T regulatory (Tregs) cells, 15 cancers were significantly correlated with CD4 memory activated Tcells, and EFHD2 was significantly correlated with common tumor-related regulatory genes such as TGF beta signaling, TNFA signaling, hypoxia, scorch death, DNA repair, autophagy, and iron death-related genes. The expression level of EFHD2 was significantly correlated with each tumor of TMB, including STAD, SARC, ACC, THYM, KICH, THCA, and TGCT. In MSI, there were significant differences in THYM, STAD, THCA, and TGCT. We used the CellMiner database to explore the sensitivity between EFHD2 gene and common antineoplastic drugs and found that the prediction of high expression of EFHD2 was related to the resistance of many antineoplastic drugs. In renal cell carcinoma, the high expression of EFHD2 is mainly concentrated in ALLOGRAFT_REJECTION, REACTIVE_OXYGEN_SPECIES_PATHWAY, INTERFERON_GAMMA_RESPONSE, IL6_JAK_STAT3_SIGNALING, INTERFERON_ALPHA_RESPONSE, and other signal pathways. GO results showed that the genes were mainly enriched in response to interferon-gamma, antigen processing and presentation, cellular response to interferon-gamma, and other pathways. KEGG results demonstrated that EFHD2 was mainly rich in phagosome, Epstein-Barr virus infection, Staphylococcus aureus infection, and other pathways. The results of Kaplan-Meier survival analysis demonstrated that the high expression of EFHD2 was significantly related to the poor prognosis.

**Conclusion:**

Our findings highlight the predictive value of EFHD2 in cancer and provide a potential research direction for elucidating the role of EFHD2 in tumorigenesis and drug resistance.

## 1. Introduction

Recent studies reveal that cancer has become a worldwide public health problem, and cancer has become the number one killer of dangerous human health [1]. In recent decades, great progress has been made in the diagnosis and treatment of cancer, especially immunotherapy based on checkpoint blockade [1]. At present, reliable prediction of biomarkers and new immunotherapy targets has attracted wide attention of scientists. EF-hand domain-containing protein D2 (EFHD2) is a conserved calcium-binding protein that is highly expressed in the immune system and central nervous system [2]. EFHD2 participates in the activation of immune cells and the regulation of immune response. The expression level of EFHD2 can influence an individual's behavior and cognitive function, such as language ability, susceptibility to motion sickness, and alcohol addiction. Moreover, EFHD2 dysfunction is linked to autoimmune and neuropathological diseases, including Parkinson's disease (PD) and Alzheimer's disease(AD) [3]. In cancer research, EFHD2 facilitates cancer cell migration and may lead to cancer metastasis [4]. Recently, some studies have found that EFHD2 promotes the epithelial-to-mesenchymal transformation (EMT) of lung adenocarcinoma and is closely related to postoperative recurrence in patients with stage I lung cancer [5]. The role of EFHD2 in cancer is getting more and more attention, but so far, the potential role and possible molecular mechanism of EFHD2 in cancer are still unclear. To date, most of the studies on EFHD2 in tumors are limited by a specific cancer type, and many studies have focused on in vitro cellular level [6]. Therefore, it is indispensable to confirm the role of EFHD2 in pan cancer [7]. In current study, our results indicated that the gene was highly expressed in 23 kinds of tumors. In addition, EFHD2 was associated with stage in many kinds of tumors. The expression of EFHD2 was closely related to the OS of 12 kinds of cancer patients. In addition, Kaplan-Meier-(KM-) plot survival analysis showed that the high expression of EFHD2 was related to the poor OS of 5 kinds of cancer, and the expression of EFHD2 was closely related to the PFS of 5 kinds of cancer patients. The expression of EFHD2 was closely related to immune infiltration, among which 18 cancers were significantly correlated with CD8 T cells, 14 cancers were significantly correlated with regulatory T cells (Tregs) cells, 15 cancers were significantly correlated with CD4 memory activated T cells, and EFHD2 was significantly correlated with common tumor-related regulatory genes such as TGFBETASIGNALING, TNFASIGNALING, hypoxia, scorch death, DNA repair, autophagy, and iron death-related genes. The expression level of EFHD2 was significantly correlated with each tumor of TMB, including STAD, SARC, ACC, THYM, KICH, THCA and TGCT. In MSI, there were significant differences in THYM, STAD, THCA and TGCT. We conducted the CellMiner database to explore the sensitivity between EFHD2 gene and common antineoplastic drugs and found that the prediction of high expression of EFHD2 gene was related to the resistance of many antineoplastic drugs. GO results showed that the genes were mainly enriched in response to interferon-gamma, antigen processing and presentation, cellular response to interferon-gamma, and other pathways. KEGG results showed that the gene was mainly rich in phagosome, Epstein-Barr virus infection, Staphylococcus aureus infection, and other pathways. The results of Kaplan-Meier survival analysis showed that the high expression of EFHD2 was significantly related to the poor prognosis of the patients.

## 2. Methods

### 2.1. TCGA Data Acquisition and Analysis

The TCGA database (https://portal.gdc.cancer.gov/), as the largest cancer gene information database, stores data including gene expression data, single nucleotide polymorphism (SNP), and copy number variation (CNV). We obtained the raw mRNA expression data and SNP data of 33 kinds of tumor data of pan cancer for follow-up analysis. The gene expression data of different tissues were downloaded from the GTEX database (https://commonfund.nih.gov/GTEx)) and then combined with TCGA data and corrected, and the differences of gene expression in different cancers were calculated. Data from each tumor cell line downloaded from the CCLE database (https://portals.broadinstitute.org/ccle/)) and the level of gene expression in these tumor tissues was analyzed according to tissue origin. In addition, the correlation between expression and tumor stage was studied.

### 2.2. Prognostic Correlation Analysis

The data of total survival time (OS) and progression-free survival (PFS) of TCGA patients were downloaded from the Xena database to further study the relationship between gene expression and prognosis. The Kaplan-Meier method was used to analyze the survival of each cancer type, and “survival” and “survminer” packages were used to evaluate the survival analysis. In addition, Cox analysis uses “survival” and “forestplot” packages to explore the relationship between gene expression and survival.

### 2.3. Analysis of Immune Cell Infiltration

The CIBERSORT algorithm was used to determine the RNA-seq data of cancer patients with different subgroups, with inferred proportion of immune infiltrating cells, and to analyze the correlation between gene expression and immune cell content. In addition, the potential relationship between gene expression and immunomodulatory factors (chemokines, immunosuppressants, immunosuppressants, MHC molecules, etc.) was explored through the TISIDB website.

### 2.4. Drug Sensitivity Analysis

The CellMiner database is based on a list of 60 cancer cells listed by the Cancer Research Center of the National Cancer Institute (NCI). The NCI-60 cell line is currently the most widely used cancer cell sample group for anticancer drug testing. In this study, NCI-60 drug sensitivity data and RNA-seq gene expression data were downloaded, and the relationship between genes and common antineoplastic drug sensitivity was discussed by correlation analysis.

### 2.5. GSVA Enrichment Analysis

Gene set difference analysis (GSVA) is a nonparametric and unsupervised method to evaluate transcriptome gene enrichment. Through the comprehensive scoring of the set of genes of interest, GSVA alters the gene level into the pathway and then access the biological function of the sample. In this study, gene sets were downloaded from Molecular Signature database (v7.0). Each gene set was scored comprehensively by GSVA algorithm, and the potential biological function changes of different samples were evaluated.

### 2.6. GSEA Enrichment Analysis

GSEA analysis uses predefined gene sets to rank genes in compliance with the degree of differential expression and then screen whether the predefined gene sets are enriched at the top or bottom of the ranking table. In this study, GSEA analysis of “clusterprofiler” and “enrichplot” packages was used to compare the differences of signal pathways between high and low expression groups of genes and to explore the possible molecular mechanism of prognostic differences among patients with 33 kinds of tumors.

### 2.7. TMB Data Analysis

TMB is defined as the total number of coding errors, insertions, base substitutions, or deletions of somatic genes detected per million bases. Therefore, the mutation frequency and the number of mutations/exon length of each tumor sample were calculated, and the TMB was defined by dividing the nonsynonymous mutation sites by the total length of the protein coding region. The value of MSI for each TCGA patient is derived from a previously published study [8].

### 2.8. Statistical Analysis

All statistical analyses were carried out in *R* language (version4.0). Univariate survival analysis was used to calculate hazard ratio (HRs) and 95% confidence interval. Kaplan-Meier analysis is used to study the survival rate of patients based on high or low levels of gene expression. All statistical tests were bilateral, and *p* < 0.05 was statistically significant.

## 3. Results

### 3.1. Analysis of Pan-Cancerous Expression of EFHD2 Gene

TCGA and GTEx datasets were employed to analyze the expression of EFHD2 in 33 human cancers. The results indicated that the gene was highly expressed in 23 kinds of tumors, including BLCA, ACC, CESC, BRCA, COAD, CHOL, GBM, ESCA, KICH, HNSC, KIRP, KIRC, LIHC, LGG, OV, LUSC, PRAD, PAAD, STAD, SKCM, UCEC, THCA, and UCS (Figure 1). In most normal tissues, the expression level of EFHD2 is lower than that in cancer tissues. Of note, the expression of EFHD2 in different tumor cell lines in CCLE expression profile is shown in the figure (Figure 2). In addition, EFHD2 is associated with stage of a variety of tumors, including CHOL, BLCA, ACC, KIRC, KICH, PAAD, LUAD, TGCT, and SKCM (Figure 3). Next, we established the relationship between the expression of EFHD2 and the prognosis of cancer patients, including OS and PFI. The results revealed that the expression of EFHD2 was closely related to the OS of 12 kinds of cancer patients, including ACC, BLCA, BRCA, KICH, KIRC, LAML, LIHC, LUAD, SKCM, STAD, THYM, and UVM tumor (Figure 4). In addition, KM-plot survival analysis uncovered that the high expression of EFHD2 was associated with five kinds of cancer OS, including ACC, KIRC, LAML, LGG, and UVM (Figure 5). The expression of EFHD2 was closely related to the PFS of five kinds of cancer patients, including ACC, BLCA, KICH, KIRC, and THYM tumor (Figure 6). Furthermore, the results of KM-plot survival analysis demonstrated that the high expression of EFHD2 was linked to the poor PFI of the three cancers, including ACC, KIRC, and THYM (Figure 7).

### 3.2. Pan-Carcinomatous Expression and Immune Infiltration

The tumor microenvironment is mainly composed of tumor-associated fibroblasts, immune cells, extracellular matrix, a variety of growth factors, inflammatory factors, special physical and chemical characteristics, and cancer cells, demonstrating that tumor microenvironment significantly affects tumor diagnosis, survival outcome, and clinical treatment sensitivity. Our results indicated that the expression of EFHD2 was closely related to immune infiltration, among which 18 cancers were significantly correlated with T cells CD8 cells, 14 cancers were significantly correlated with T cells regulatory (Tregs) cells, and 15 cancers were significantly correlated with T cells CD4 memory activated cells (Figure 8). We further analyzed the tumor microenvironment of renal cell carcinoma (KIRC). The results showed that the scores of TMEscore, CD_8_T_effector, Immune_Checkpoint, Antigen_processing_machinery, TMEscoreA, Mismatch_Repair, Nucleotide_excision_repair, DNA_damage_response, DNA_replication, Base_excision_repair, Pan_F_TBR, EMT2, and EMT3 were significantly correlated with renal cell carcinoma (Figure 9).

### 3.3. Pan-Carcinomatous Expression and Key Regulatory Genes

In this section, gene coexpression analysis was carried out to explore the relationship between EFHD2 expression and 33 tumor immunity-related genes. The analyzed genes included MHC, immune activating factor, immunosuppressive factor, chemokine, and chemokine receptor protein. The results indicated that almost all immune-related genes were significantly associated with EFHD2 (Figure 10). In addition, EFHD2 was significantly associated with tumor-related regulatory genes such as TGF beta signaling, TNFA signaling, hypoxia, scorch death, DNA repair, autophagy, and iron death-related genes (Figure 11).

### 3.4. Pan-Carcinomatous Expression and TMB and MSI

TMB and MSI are two new biomarkers related to immunotherapy response. The purpose of this study was to explore the relationship between the expression of EFHD2 and TMB. The results portended that the expression level of EFHD2 was significantly correlated with each tumor of TMB, including STAD, SARC, ACC, THYM, KICH, THCA, and TGCT (Figure 12). In MSI, there were significant differences in gene EFHD2 among THYM, STAD, THCA, and TGCT (Figure 13).

### 3.5. Pan-Cancer Expression and Drug Sensitivity

We conducted the CellMiner database to explore the sensitivity between EFHD2 gene and common antineoplastic drugs and further calculated the correlation between the gene expression and drug IC50. It was found that the high expression of gene EFHD2 was associated with multiple antineoplastic drug resistance (Figure 14). Among them, EFHD2 was negatively correlated with fulvestrant, acetalax, bisacodyl, active ingredient of viraplex, SR16157, and lapatinib and positively correlated with azacitidine, irinotecan, uracil mustard, triapine, pralatrexate, triethylenemelamine, perifosine, gemcitabine, mitomycin, floxuridine, thiotepa, midostaurin, and staurosporine.

### 3.6. Pan-Cancer Expression and GSVA/GSEA

In order to further study the molecular mechanism of EFHD2 gene in pan cancer, we first scored all tumors with GSVA, and then in each tumor, using the median of gene expression, the samples were divided into high and low expression groups for comparison. The results revealed that in renal cell carcinoma, the high expression of EFHD2 was mainly concentrated in ALLOGRAFT_REJECTION, REACTIVE_OXYGEN_SPECIES_PATHWAY, INTERFERON_GAMMA_RESPONSE, IL6_JAK_STAT3_SIGNALING, INTERFERON_ALPHA_RESPONSE, and other signal pathways (Figure 15). The GSEA analysis of EFHD2 and renal cell carcinoma is presented in the figure (Figure 16).

### 3.7. WGCNA Analysis

Based on the expression profile data of KIRC, we further construct the WGCNA network and explore the EFHD2-related coexpression network in KIRC. The soft threshold *β* is determined by the function “powerEstimate,” and the soft threshold is set to 9. Based on the tom matrix detection gene module, a total of 11 gene modules were detected in this analysis. They are black, blue, brown, green, greenyellow, grey, megenta, red, tan, turquoise, and yellow. Through further analysis between modules and traits, we found that MEmagenta modules had the highest correlation (cor = 0.68, *p* = (1*e*/77)) (Figure 17). We further conducted the magenta module gene for pathway analysis, and GO results revealed that the gene was mainly enriched in response to interferon-gamma, antigen processing and presentation, cellular response to interferon-gamma and other pathways (Figure 18). Furthermore, KEGG demonstrated that the EFHD2 mainly enriched phagosome, Epstein-Barr virus infection, Staphylococcus aureus infection, and other pathways (Figure 19).

### 3.8. Analysis of Risk and Independent Prognosis of EFHD2

We construct the nomogram prediction model according to the EFHD2 expression and clinical symptoms and reveal their results through regression analysis in the form of line chart, in which the results of logical regression analysis show that in our KIRC samples, the prediction efficiency of the EFHD2 gene expression for the model is presented in the figure (Figure 20). In addition, this study draws correction curves for three and five years at the same time, and the model effect is consistent (Figure 21).

### 3.9. EFHD2 and Immunotherapy

In this section, we download the data set of PD-1 immunotherapy for clear cell renal cell carcinoma tumors (Braun 2020, Nat Med). A total of 181patients who received nivolumab therapy with complete survival information were included. The results of Kaplan-Meier survival analysis showed that the high expression of EFHD2 was significantly correlated with poor prognosis (Figure 22).

## 4. Discussion

Our results revealed that EFHD2 was highly expressed in 23 kinds of tumors, including ACC, BLCA, BRCA, CESC, CHOL, COAD, ESCA, GBM, HNSC, KICH, KIRC, KIRP, LGG, LIHC, LUSC, OV, PAAD, PRAD, SKCM, STAD, THCA, UCEC, and UCS. So far, there is little literature on the prognostic value of EFHD2 in cancer patients. In our current study, the expression of EFHD2 was closely related to the OS of 12 kinds of cancer patients, including ACC, BLCA, BRCA, KICH, KIRC, LAML, LIHC, LUAD, SKCM, STAD, THYM, and UVM tumors. In addition, the expression of EFHD2 was closely related to the PFS of five kinds of cancer patients, including ACC, BLCA, KICH, KIRC, and THYM tumors. The results of KM-plot survival analysis showed that the high expression of EFHD2 was associated with three cancerous PFS, including ACC, KIRC, and THYM, suggesting that EFHD2 may have the potential to indicate the malignant degree and prognosis of the tumor.

It is well acknowledged that the emergence of EMT renders cancer cells that have mesenchymal phenotype and stem cell-like characteristics; so, they have invasiveness and chemotherapy resistance [9]. Our analysis of EMT-related genes further supports the carcinogenic and dry-related role of EFHD2 in cancer. MSI and TMB have attracted much attention recently, and they are considered as promising biomarkers for predicting the efficacy of immunotherapy [10]. Our results indicated that the expression level of EFHD2 was significantly correlated with each tumor of TMB, including STAD, SARC, ACC, THYM, KICH, THCA, and TGCT. In MSI, there were significant differences in gene EFHD2 in THYM, STAD, THCA, and TGCT. These results strongly suggest that the expression of EFHD2 may affect the response of cancer patients to immune checkpoint therapy, which will provide new clues for the prognosis of immunotherapy. Therefore, cancer patients with low expression of EFHD2 and high levels of MSI and TMB are more likely to benefit from immunotherapy.

Tumor microenvironment significantly influences tumor diagnosis, survival outcome, and clinical treatment sensitivity; so, the relationship between gene expression and microenvironment has become the focus of cancer research in recent years [11, 12]. Our results showed that the expression of EFHD2 was closely related to immune infiltration, among which 18 cancers were significantly correlated with T cells CD8 cells, 14 cancers were significantly correlated with T cells regulatory (Tregs) cells, and 15 cancers were significantly correlated with T cells CD4 memory activated cells. We further analyzed the tumor microenvironment of renal cell carcinoma (KIRC). The results showed that the scores of TMEscore, CD_8_T_effector, Immune_Checkpoint, Antigen_processing_machinery, TMEscoreA, Mismatch_Repair, Nucleotide_excision_repair, DNA_damage_response, DNA_replication, Base_excision_repair, Pan_F_TBR, EMT2, and EMT3 were significantly correlated with renal cell carcinoma. The above results suggest that EFHD2 is significantly involved in the regulation of immune cells, especially killer T cell infiltration, and the intervention targeting EFHD2 will provide a good basis for improving the efficacy of patients and immunotherapy.

At present, the correlation between gene expression and drug resistance has been very clear [13, 14]. Our study found that the high expression of gene EFHD2 is associated with a variety of antineoplastic drug resistance. Therefore, EFHD2 may be used as a good target to predict tumor chemosensitivity in the future. In addition, the role of EFHD2 in tumor immune microenvironment is still unclear and needs to be confirmed by further research. According to the immune cell estimation algorithm, the correlation between the expression of EFHD2 and the content of immune cells may be related to the type of tumor. Download the data set of PD-1 immunotherapy for clear cell renal cell carcinoma (ccRCC), and the results of Kaplan-Meier survival analysis indicated that the high expression of EFHD2 was significantly correlated with poor prognosis. We speculate that the immune checkpoint gene is positively correlated with the expression of EFHD2 in most tumor types, suggesting that EFHD2 may be involved in immune escape. Therefore, it is necessary to further study the relationship between EFHD2 expression and immune infiltration in vitro and in vivo [12]. In addition, our GSEA analysis showed that in renal cell carcinoma, the high expression of EFHD2 was mainly concentrated in ALLOGRAFT_REJECTION, REACTIVE_OXYGEN_SPECIES_PATHWAY, INTERFERON_GAMMA_RESPONSE, IL6_JAK_STAT3_SIGNALING, INTERFERON_ALPHA_RESPONSE, and other signal pathways. Therefore, we believe that EFHD2-mediated signal pathways play an important role in the progression of cancer.

The significance of our current study is that the multifaceted functions of EFHD2 were implicated in cancer, which not only further confirmed the previous results of EFHD2 but also give the potential to corroborate the function modulate by EFHD2 in the tumor drug resistance, immunotherapy, and microenvironment. Since our study acts as a comprehensive bioinformatics analysis on the basis of multiple databases, there are several inevitable limitations. First of all, our results are based on the prediction of bioinformatics data, rather than experimental confirmation; so, further molecular biology experiments are needed to verify [15]. Secondly, our results are mainly reflected in the analysis of mRNA expression of EFHD2. As the direct executor of biological function, the analysis based on EFHD2 level will make the results more convincing. In addition, our study only made correlation analysis, but the molecular mechanism of EFHD2 in tumor dryness and immune infiltration needs to be further studied. Based on the above, our pan-cancer analysis systematically discussed the characteristics of EFHD2 from many aspects, such as expression, survival prognosis, gene mutation, tumor immune microenvironment, and drug resistance. We conclude that EFHD2 may be a potential target for tumor therapy considering that it is abnormally expressed in many cancers and predicts a poor prognosis of cancer patients. Meanwhile, we observed the frequent amplification of EFHD2, and the expression of EFHD2 was positively correlated with amplification. In addition, the abnormal expression of EFHD2 is linked to the immunotherapy-related genes and tumor microenvironment of different types of tumors. In addition, it should be pointed out that EFHD2, as a potential drug resistance target, can predict the sensitivity of tumor cells to chemotherapeutics. Therefore, our study provides a new basis for elucidating the potential role of EFHD2 in tumorigenesis, drug resistance, and immunotherapy. Finally, our results also point out the potential direction for further elucidating the function of EFHD2 in cancer in the future.

## Figures and Tables

**Figure 1:** The general situation of the expression of single gene in TCGA and GTEX pan-cancerous tissues. In 33 kinds of tumors, the difference of single gene between tumor and normal tissue was analyzed, among which yellow was tumor tissue and blue was normal tissue.

**Figure 2:** The expression of this gene in CCLE tumor cell line. Different colors represent different tumor cell lines (visualization: ggplot2 and ggpubr package).

**Figure 3:** The relationship between gene expression and tumor stage. In 33 kinds of tumors, the differences of genes in samples of different stages were analyzed (ggpubr package).

**Figure 4:** According to the gene median value, the patients were divided into the high-risk group and low-risk group. Using Kaplan-Meier to analyze the survival of pan-cancer tissues (survival package), there was a significant difference when the *p* value was less than 0.05. Red is the high expression group, and blue is the low expression group.

**Figure 5:** The univariate Cox regression analysis (forestplot package) of the gene in pan-cancer tissues showed that the *p* value was less than 0.05. There was a significant difference between the two groups. HR > 1 is a risk factor, and HR < 1 is a protective factor.

**Figure 6:** The univariate Cox regression analysis (forestplot package) of the gene in pan-cancer tissues showed that the *p* value was less than 0.05. There was a significant difference between the two groups. HR > 1 is a risk factor, and HR < 1 is a protective factor.

**Figure 7:** According to the gene median value, the patients were divided into the high-risk group and low-risk group. Using Kaplan-Meier to analyze the survival of pan-cancer tissues (survival package), there was a significant difference when the *p* value was less than 0.05. Red is the high expression group, and blue is the low expression group.

**Figure 8:** The TIMER database was used to calculate the immune cell infiltration information of each tumor. The heat map can be used to show the association between the immune infiltration and the target gene in pan cancer. Red indicates positive correlation, and blue indicates negative correlation (visualization using ggplot2, ggpubr, patchwork, and showtext packages).

**Figure 9:** The immune cell content of each patient was quantified by the CIBERSORT algorithm, and the correlation between gene expression and immune cell content was analyzed. Red represents the group of high gene expression, and yellowish green represents the group of low gene expression.

**Figure 10:** Analysis of the correlation between genes and immune activation genes. In different cancers, the correlation between genes and immune-activated genes was analyzed, in which red represents a positive correlation and blue represents a negative correlation.

**Figure 11:** Analysis of the correlation between genes and immune activation genes. In different cancers, the correlation between genes and immune-activated genes was analyzed, in which red represents a positive correlation and blue represents a negative correlation.

**Figure 12:** The correlation between the expression of this gene and TMB in pan cancer. The blue of the inner circle was the low expression group, and the red of the outer circle was the high expression group (use fmsb, limma, and dplyr packages for analysis).

**Figure 13:** The correlation between the expression of this gene and TMB in pan cancer. The blue of the inner circle was the low expression group, and the red of the outer circle was the high expression group (use fmsb, limma, and dplyr packages for analysis).

**Figure 14:** The correlation diagram with the IC50 of the drug. The correlation map between the gene and the IC50 of the drug and the slope of the straight line are the correlation coefficient between the gene and the drug.

**Figure 15:** Enrichment analysis of single gene pan-cancer-related GSVA pathway. The blue part represents the high expression group enrichment pathway, and the green part represents the low expression group enrichment pathway (use GSVA and limma packages for analysis).

**Figure 16:** Enrichment analysis of single gene pan-cancer-related GSEA pathway. The blue part represents the high expression group enrichment pathway, and the green part represents the low expression group enrichment pathway (use GSEA and limma packages for analysis).

**Figure 17:** Analysis of the correlation between module and gene expression/clinical symptoms. The upper number is the correlation coefficient, and the lower number is the *p* value.

**Figure 18:** Analysis of GO/KEGG enrichment pathway of the most correlated modular genes.

**Figure 19:** Analysis of GO/KEGG enrichment pathway of the most correlated modular genes.

**Figure 20:** The line diagram related to the model and different peers represent the different clinical characteristics of the samples.

**Figure 21:** The correction curve of the model correlation line chart, five years in blue and eight years in red.

**Figure 22:** According to the gene median value, the patients were divided into the high-risk group and low-risk group. Using Kaplan-Meier to analyze the survival of pan-cancer tissues (survival package), there was a significant difference when the *p* value was less than 0.05. Red is the high expression group, and blue is the low expression group.

## Data Availability

No data were used to support this study.
